The article "Evaluation of Upper Limb Muscle Activation Using Musculoskeletal Model with Wearable Assistive Device" was published in 2022. Journal: Appl Bionics Biomech.

# Evaluation of Upper Limb Muscle Activation Using Musculoskeletal Model with Wearable Assistive Device

**DOI:** 10.1155/2022/8908061

**Published:** 2022-07-06

**Authors:** M. F. Ashari, A. Hanafusa, S. Mohamaddan

**Affiliations:** Department of Bioscience and Engineering, Shibaura Institute of Technology, 337-8570 Saitama, Japan

## Abstract

In recent years, wearable assistive device has been used to support upper arm movement training for rehabilitation purposes. A wearable assistive device could affect the muscle output during motor tasks to support upper limb disorder rehabilitation training. However, the investigation of muscle activity with the given assistive force is not widely investigated. In this study, the evaluation of upper limb muscle activities using musculoskeletal simulation systems with the developed wearable cable-driven assistive device has been carried out. An experimental protocol consisting of a series of motions was executed with five healthy subjects. Muscle activation on the brachioradialis, biceps, and triceps muscles was measured by using surface electromyography (EMG) and analyzed. The simulations with a musculoskeletal model to estimate muscle output with and without a wearable assistive device were performed for three tasks. An assistive upper arm device was integrated into the musculoskeletal model, and the desired assistive force is translated to the arm joint along with a tendon routing structure. Assisting movement by the wearable device was evaluated by measuring muscle activation with-assist and without-assist conditions. The results show that the use of the wearable assistive device can effectively assist in arm movement. Comparisons of measured EMG muscle data and the musculoskeletal model revealed that muscle force was generated throughout the arm. The integrated musculoskeletal model results show that muscle force values for two primary muscles (biceps and brachioradialis) were reduced during the simulated task when wearing the assistive device. These results are congruent with expectations, with the assistive device that supports the upper limb movement, providing practical assistance. The results highlight the importance of evaluating muscle output for the developed wearable assistive device to support the assistive movement. Lastly, the musculoskeletal simulation system could reduce the resource-intensive, and time consumed with the experimental testing could be achieved.

## 1. Introduction

In the past years, in many areas, assistive devices have been developed to support humans in performing different types of tasks and support activity of daily life. Assistive devices have also been developed in the medical or rehabilitation field. These devices treat or support patients in case of loss of function caused by diseases, especially stroke patients.

The article "Evaluation of Upper Limb Muscle Activation Using Musculoskeletal Model with Wearable Assistive Device" was published in 2022. Journal: Appl Bionics Biomech.

Stroke often causes permanent and complex long-term disability in adults, reducing the patients' quality of life and bringing enormous pain to their physiology and psychology and burdening families in general [1, 2]. In literature, upper limb hemiparesis is widely reported as one of the primary impairments after stroke. While many patients recover ambulatory function after dense hemiplegia, arm motor skills restoration is often incomplete. More than 60% of patients cannot use their paretic hands in functional activities [3]. The recovery of arm movements is one of the most important goals during stroke rehabilitation to avoid long-term disability that may restrict activities of daily living (ADL) and social and occupational activities and lead to depression.

Effective rehabilitation training can improve patients' nerve function and maintain the degree of joint activity to help the patient gain their upper limb function capability. Traditional rehabilitation training is a one-to-one auxiliary exercise for patients by therapists. This method is challenging to develop an effective treatment plan, and it is tough to control accurately [4]. The traditional treatment methods, which are based on the therapist's clinical experience, also have significant staff consumption problems, long rehabilitation cycles, limited rehabilitation effects, and so on. With rehabilitation assistive technology and medicine development, the rehabilitation device has become a novel assistive rehabilitation treatment technology. It is essential to utilize technology for rehabilitation training to recover stroke patients' limb function [5]. The research and application of rehabilitation device systems are expected to effectively alleviate the contradiction between the supply and demand of rehabilitation medical resources and improve the quality of life of stroke patients [5, 6].

The wearable assistive device that applies forces to the body to assist with motor tasks is one approach that may assist people during the rehabilitation of upper limb disorder. For example, exoskeletons could improve task economy [7], enhance strength and functional ability [8, 9], lower biomechanical loads and associated injury risks [10], or protect healing musculoskeletal tissues during recovery from trauma surgery. At present, a variety of exoskeleton rehabilitation robots are developed, e.g., a dynamic exoskeleton system ADEN-7 robot with 7 degrees of freedom [11] and ARMIN robot with six degrees of freedom (four active and two passive) semiexoskeleton structure [12], an ARMEO robot providing arm weight reduction support system for training, enhancing performance feedback and evaluation tools [13]. Currently, it is a relatively safe and efficient rehabilitation robot structure. However, most of these high-technology devices are placed at the rehab center and need to be operated on by specialists and the patient to come regularly. Therefore, it is crucial to investigate the potential of adapting this technology which is potentially lighter, more affordable, and more convenient to use (e.g., basic operating manual) than high technology exoskeletons. These attributes make the assistive device more wearable and suitable for continuous use at the home, workplace, and community.

The article "Evaluation of Upper Limb Muscle Activation Using Musculoskeletal Model with Wearable Assistive Device" was published in 2022. Journal: Appl Bionics Biomech.

When providing effective assistance, it is expected that wearable assistive devices can reduce muscle output (e.g., muscle activations) during motor tasks. Experimental testing has provided a necessary direct evaluation of muscle output for powered [9, 14] and passive [9, 15–17] exoskeletons. However, experiments are resource-intensive and possibly require several iterations of physical prototypes. Especially in the early design of human-machine interfaces, computational musculoskeletal modeling and simulation tools have offered a cost-effective, alternative approach to experimental testing for both upper extremities [18, 19] and lower extremity exoskeletons [20]. Thus, in the proposed study, we used computational modeling and simulation to evaluate muscle output during dynamic right upper limb movements for a wearable assistive device we have developed to assist with right upper limb movement. Our study's primary goal was to quantify muscle output with and without our wearable assistive device during three simulated tasks involving dynamic right upper limb movement. We hypothesized that the resulting exoskeleton output force would cause muscle output to be lower for some muscles with the assistive device than without wearing the device.

## 2. Materials and Methods

### 2.1. Assistive Device

Owing to the anatomy theory, motion mechanism, and range of human upper limbs for rehabilitation training, a wearable assistive device with a combination of servo motor and cable mechanism was developed. This device can generate elbow flexion and extension movement motions by pulling the cable hung on a pulley connected to the forearm part. A cable-driven motor is rear-mounted to achieve long-distance transmission and reduce the drive inertia of the end joints. The mechanism and details of the device can be referred to in this paper [21]. The shoulder joint internal/external rotation mechanism's transmission mechanism is an active gear with belt transmission, where both ends of the maximum reachable range are provided with a limiter switch. Once it exceeds the rehabilitation range, the passive gear will be blocked. It cannot continue to move, ensuring the subject's safety and avoiding secondary injuries to the subject.

The article "Evaluation of Upper Limb Muscle Activation Using Musculoskeletal Model with Wearable Assistive Device" was published in 2022. Journal: Appl Bionics Biomech.

As illustrated in Figure 1 above, the elbow motion mechanism is constructed by a two-way winding coil structure. The driven part of the elbow joint movement mechanism is mounted on the forearm. The two-way driven pulley of the motor transmits the power to the elbow through the cable; thus, it completes the elbow flexion/extension motion. The wearable device's range of motion and its operational degree of freedom is shown in Figure 2.

As mentioned in this study's objective, the relationship between the assistive force given by the assistive device and its relationship to the muscle output will be investigated further. Therefore, an experimental procedure has been conducted to measure the assistive force during the device's upper limb motion. Three specified tasks—elbow flexion and extension, shoulder flexion and extension, and inner rotation with shoulder flexion and extension—have been designed according to the device's capability and also associated with the training in rehabilitation upper limb movements. A load cell (TCS-20L, NEC company, Japan) has been used to measure the tension force generated from the cable during the power transmission for the movements. The measurement setting is connected to the motion capture system so that every activity with the subject is recorded simultaneously.

## 3. Experimental Protocol

An experimental protocol was approved by the Shibaura Institute of Technology (SIT) Review Board. All subjects were told the aim of the experiments and provided written consent to participate in this study, and this consent procedure was approved by SIT. The individual in this manuscript has given written informed consent to publish these case details. In this study, five right-handed able-bodied subjects (all males, ages ranging 23-30-year old; weight 58.2 ± 6.8 kg; height 167 ± 6.2 cm) participated. The subjects did not have any skeletal or muscular diseases that could affect their muscle activity. The protocol involved performing three motions with two conditions which were with and without wearing the assistive device. The assistive device was applied to the subjects in the right arm. The arm movement speed is naturally moved according to the subjects without the device. When using the device, the speed of the movement liaises with the speed of the motor used.

During the experiment, the subjects were quietly seated in the chair with their torso keeping upright and their right hand keeping relaxing. Three motions shown in Figures 3–5 are designed to obtain the motion of the right upper limb. The traces in every figure indicated the movement trajectory from the initial position to the destination position in a single trip of each motion and returned to the initial position. These arm movements are freely repeated to capture the commonality and the EMG and motion properties' variability.

The article "Evaluation of Upper Limb Muscle Activation Using Musculoskeletal Model with Wearable Assistive Device" was published in 2022. Journal: Appl Bionics Biomech.

## 4. Experimental Setup

### 4.1. Motion Recording

Data were acquired in the Shibaura Institute of Technology (SIT) laboratory using the 3D Motion Capture System. This equipment consists of infrared cameras, which can capture the 3D position of the different markers over time. Ten markers are placed in the subject to capture the different motions analyzed. The markers' numbers and locations were selected following the International Society of Biomechanics (ISB) recommendations based on body landmarks to place the markers. Finally, since only the motion of the right arm is studied, the markers are only set in the right part of the body, and the device was also applied to the subjects at the right shoulder. The markers setup is shown in Figure 6, with the corresponding names in Table 1.

### 4.2. Electromyography (EMG) Measurement

Surface EMG signals were acquired by a commercial EMG acquisition system (P-EMG plus, http://oisaka.co.jp, Japan). In this experimental setup, the configuration of the EMG recording is shown in Figure 7. Three predominant muscles activating the elbow DoFs were selected to be the test's muscles: biceps, triceps, and brachioradialis muscle. Eight channels (only three channels were used) of the bipolar differential amplifier were carefully placed on these muscles according to the anatomy and hand touch experience according to the SENIAM guide. The skin underneath the electrodes was cleaned with an alcohol patch to reduce the skin's and sensors' resistance. The active EMG electrodes of each channel were positioned at the muscle belly along the muscle fiber direction with the reference electrode orthogonal to the active electrodes' midline. The ground electrode was attached to the elbow bone. The subjects were weighted with a 1 kg load strapping on the right wrist for every motion. EMG signals were recorded in each posture at 1 kHz that were digitally filtered using a bandpass filter (20 to 500 Hz) in addition to a notch filter. The raw EMG was rectified, and the RMS EMG was computed for the test's most stable region.

### 4.3. Musculoskeletal Model

The dynamic upper extremity musculoskeletal model [23], as shown in Figure 8, had four rigid segments representing the rib cage and right humerus, radius, and hand. The model was modified to include only 32 Hill-type muscle-tendon actuators. For our simulations, we limited the dynamic model to 4 degrees of freedom: shoulder elevation, elevation plane angle of the shoulder, axial shoulder rotation, and elbow flexion. The other upper extremity degrees of freedom, such as wrist flexion, wrist deviation, and forearm rotation, were held constant at an angle of 0*°*. The fingers' movement and the wrist are not studied for two reasons: the considered arm support will not articulate the fingers, and those are the last part affected by the disease.

The article "Evaluation of Upper Limb Muscle Activation Using Musculoskeletal Model with Wearable Assistive Device" was published in 2022. Journal: Appl Bionics Biomech.

### 4.4. Upper Arm-Device Integrated Model

The model of the device was created previously using CREO software. These 3-dimensional elements representing the 3 main parts of the device, the trunk, upper arm, and lower arm, as shown in Figure 9(a), were added to the musculoskeletal model in OpenSim. The mass of each component was defined according to the materials for developing the device. The moments of inertia were estimated from the computer-aided design model according to the defined materials. During this integration to build a human-device model, the new weight consists of body and device weight, calculation center of mass, and inertial parameters are already considered, and the effect is realized during the simulation.

### 4.5. Analysis of the Effect of the Assistive Force on Muscle Activation Using Biomechanical Simulations

We simulated tasks with and without the assistive device to evaluate the muscle output from the given force measured in the experiments. As explained previously, joint kinematics were defined from the experimentally measured healthy upper limb movement subjects. To carry out muscle analysis, the Computed Muscle Control (CMC) Tool was solved to compute a set of muscle activations required for the dynamic model to track the desired kinematics by minimizing the sum of muscle activations [16] In this study, the effect of the assistive force on the muscle output was evaluated. The acquired assistive force from the experimental was defined in OpenSim and applied to the integrated human-device model system to acquire the interested muscle activations to support the arm movement.

## 5. Results

We compared the steady-state muscle activations between simulations with and without the assistive device for the simulated static task. For each of the three simulated dynamic upper limb movements, we computed an outcome measure of the muscle activity for each muscle of interest (brachioradialis, biceps, and triceps). The muscles' location is shown previously in Figure 7.

### 5.1. Upper Limb Motion: 90-Degree Elbow Flexion and Extension

The result of the experiments and simulations are presented. Figures 10–12 compare three interested muscles for the upper limb movement with and without wearing the assistive device. Experiments on the upper arm device had shown that muscle activations could be significantly reduced when assistive force was enabled during upper limb movements. Overall, the results show that each of the muscles activated reduced thanks to the presence of the assistive device. In Figure 10 above, the most significant activated muscle would be brachioradialis (green), which can be observed in EMG measured and simulation data from force produced. The initial peaks are mainly visible during the elbow's flexion (within the first 40% of movement) both in experimental and simulation for brachioradialis and biceps muscle. As reported in [24–26], the primary activated muscle for elbow flexion movement would be in brachioradialis and biceps muscles, and the result from the EMG could confirm the reported article. However, we can see the visible peak when the arm is in extension motion (the last 50% of the movement) for the brachioradialis muscle. This is because the muscle was trying to sustain the movement because of the 1 kg weight worn by the subject on the wrist. On the other hand, we could observe the significant triceps muscle peak during the extension motion in musculoskeletal simulation with and without wearing the device. The triceps muscle is an extensor muscle of the upper extremity. Positioning and EMG sensor attachment probably cause minimal detection for the triceps muscle area during the experiment.

The article "Evaluation of Upper Limb Muscle Activation Using Musculoskeletal Model with Wearable Assistive Device" was published in 2022. Journal: Appl Bionics Biomech.

### 5.2. Upper Limb Motion: Maximum Shoulder Flexion and Extension

The result in Figure 11 shows a similar group of muscles activated during the arm's flexion, which peaks in the brachioradialis, and biceps muscles can be observed in both experiment and simulation data for the first 40% of the movement. Then, these muscles also have another activation during the shoulder flexion. Although commonly, the muscle involved during elbow flexion is mainly at the shoulder, the weight in the subject's arm could cause the muscle to do extra work to sustain the shoulder and arm during the shoulder flexion. Only the initial peak for both muscles can be observed when the subject wears the device. Due to the assisted movement by the device, the elbow and shoulder are well supported during the shoulder flexion, and extension movement causes no muscle activated during the motions. In both experiments, low detection would probably be from the poor sensor attachment and the excessive fat region for triceps muscle data.

### 5.3. Upper Limb Motion: Inner Elbow Flexion and Extension

For inner elbow flexion and extension, the shoulder muscle would be the most anticipated during these movements according to the muscle anatomy of the upper limb human movement. However, since this is a preliminary evaluation, we only focus on three muscles for all the motions for comparison, and none of the shoulder muscles is evaluated. Overall results in Figure 12 show that a shallow muscle peak is activated across the muscles. This visible activated muscle may be because of the muscle trying to hold or sustain the arm with the weight during the motion.

The article "Evaluation of Upper Limb Muscle Activation Using Musculoskeletal Model with Wearable Assistive Device" was published in 2022. Journal: Appl Bionics Biomech.

## 6. Discussion

Wearable assistive devices can potentially offset substantial arm loading during upper limb movement tasks. This study compared the functionality of the assistive device developed in this study for upper arm dynamic movements and its effect on the muscle output. Together with the experimental condition, two computer-based musculoskeletal models with and without device parameters have been set up. Specifically, we used measured tension forces during the device motion as input to compare differences in force and activation in the right arm muscles (Brachioradialis, biceps, and triceps) activity.

Results showed that a musculoskeletal model with and without an integrated assistive device could produce muscle activation patterns similar to the EMG measured for all muscles of interest during the simulated upper dynamic tasks. A comparison of measured EMG muscle data and human-device models revealed that, although the model did not fully incorporate similar muscle physiology completely, muscle force was generated throughout the arm comparable with measured muscle activity from the experimental. The integrated human-device model produced encouraging results such that muscle force values for 2 primary muscles (biceps and brachioradialis) were reduced during the simulated task when wearing the assistive device. These results are congruent with expectations, with the assistive device manages to support the upper limb movement, providing practical assistance.

Our study has several assumptions and limitations. Firstly, only healthy subjects were tested and modeled in this study, and the findings may not reflect those of an affected upper limb due to the stroke disease. Secondly, differences in kinematics between the assistive device joints and the anatomical upper limb joints may have influenced model calculation during the simulation. However, they are unlikely to have influenced the main finding in this study of evaluation of significantly reduced muscle output when wearing the assistive device. Even though our simulation results are based on our developed assistive device design, our main findings are generalizable to other wearable devices, including cable-driven ones.

The article "Evaluation of Upper Limb Muscle Activation Using Musculoskeletal Model with Wearable Assistive Device" was published in 2022. Journal: Appl Bionics Biomech.

We only simulated 3 specific upper extremity movements in the present study that capture a small subset of possible upper arm movements. A more significant number of movements representing the wide variety of daily living tasks should be evaluated in the future to determine the effect of the assistive device more comprehensively on user biomechanics. In addition, we constrained all simulations and conditions to the same experimental kinematics from the healthy subject who was not impaired and did not use the device in regular daily life. Someone using an assistive device regularly may adapt their movement, as shown for other passive devices [26].

Our developed assistive device's primary function is to help with ADL tasks for patients who cannot move one arm. However, the capability of the assistive device to assist the arm movement and its effect on muscle activity has not been studied to date. This study demonstrated that upper limb movement assisted by the wearable assistive device could reduce peak muscle force confirming the study hypothesis.

## 7. Conclusions

To successfully translate wearable assistive technology to upper limb disability patients during rehabilitation training, it is critical to understand its effectiveness, usability, and biomechanical interaction with humans. As a first step toward accomplishing this goal, we quantitatively evaluated our developed assistive device's mechanical and biomechanical performance. Our results showed that the device could reduce the muscle activity of several muscles crossing the upper arm. However, our mechanical evaluation revealed aspects of the design that limit the assistive device's assistance. In our future work, different assistance levels and identifying a range of assistance that most enhances arm motor function and biomechanics will be explored further. More comprehensive biomechanical studies will be performed to assess the device for more biomechanical parameters (e.g., joint kinematics), more participants (both able-bodied subjects and people with upper arm disability), and more movements that typify activities of daily living. Finally, several design refinements need to be made, especially those that reduce friction and add a motion range to the system.

The method's limitations suggest that if the interest is focused on muscle forces, EMG data can only provide a preliminary assessment of muscle activation patterns and does not provide information on how muscle forces change within specific tasks due to the nonlinear relationship between EMG and muscle forces [27]. The ideal way to compare the results of a musculoskeletal model and actual internal structure forces would be to measure joint reaction forces during the movement of interest and relate them to the calculated joint reaction forces. This type of validation is limited to impaired participants, who might not even complete all tasks.

The article "Evaluation of Upper Limb Muscle Activation Using Musculoskeletal Model with Wearable Assistive Device" was published in 2022. Journal: Appl Bionics Biomech.

Furthermore, the musculoskeletal models were not adjusted participant specifically in the current study, further explaining the differences between the model predictions and the EMG measurements. However, it can be assumed that the participant-specific differences based on the available treatment are substantially averaged out over the five participants. Moreover, the goal was to assess whether this human-device integrated model can be used in future research for evaluating muscle output during rehabilitation training when using the assistive device. To conclude, this study showed that the integrated human-device musculoskeletal model yielded good agreement between the measured and estimated muscle activity for most conditions and muscles. Therefore, it can be used for further analysis in similar groups of participants.

## Figures and Tables

**Figure 1:** The overview of the developed wearable assistive device [22] and the load cell position for tension force measurement.

**Figure 2:** Assistive device motion range according to its degree of motion.

**Figure 3:** Subjects wearing an assistive device were asked to flex their elbow close to 90 degrees and return to the initial position. Data (b) shows measured elbow flexion angle and tension force versus time.

**Figure 4:** Subject wearing an assistive device performing maximum shoulder flexion and extension. This movement acquires the subject to flex the elbow to the close to 90 deg, and then the upper arm will be brought to the upper limit of the arm's reachable motion and then return to the initial position. Data (b) shows measured elbow flexion angle, shoulder flexion angle, and tension force versus time.

**Figure 5:** Subject wearing an assistive device performing maximum shoulder flexion and extension to the initial position. The arm's initial position was kept in front of the inner side of the frontal body of the subject. The elbow was flexed to the maximum and returned to the initial position. Data (b) shows measured elbow flexion angle, shoulder flexion angle, and tension force versus time.

**Figure 6:** Ten marker locations following the International Society of Biomechanics (ISB).

**Figure 7:** EMG signals were recorded from sets of electrodes attached to the muscles of interest (biceps, triceps, and brachioradialis), while the subjects were weighted with a load on the wrist.

**Figure 8:** Dynamic musculoskeletal model of the upper limb. The dynamic model incorporates 7 degrees of freedom, including shoulder rotation and elevation and wrist flexion, wrist deviation and elbow flexion, and elevation plane of the shoulder and forearm rotation.

The article "Evaluation of Upper Limb Muscle Activation Using Musculoskeletal Model with Wearable Assistive Device" was published in 2022. Journal: Appl Bionics Biomech.

**Figure 9:** Wearable device model components and their position and orientation in the model. The modeled components shown in (a) were designed using the CAD Creo Software and later been imported into the OpenSim software to produce a human-device integrated model (b) that will later be used in simulation in the OpenSim software.

**Figure 10:** Comparison of EMG from experimental and muscle activations computed from OpenSim resulting in three muscle force brachioradialis (green), biceps (magenta), and triceps (blue) for 90-degree elbow flexion and extension motion with and without the assistive device.

**Figure 11:** Comparison of EMG from experimental and muscle activations computed from OpenSim resulting in three muscle force brachioradialis (green), biceps (magenta), and triceps(blue) for maximum shoulder flexion and extension motion with and without the assistive device. ∗∗ (Flex: flexion; S. Flex: shoulder flexion; Ext: extension).

**Figure 12:** Comparison of EMG from experimental and muscle activations computed from OpenSim resulting in three muscle force brachioradialis (green), biceps (magenta), and triceps (blue) for inner elbow flexion and extension motion with and without the assistive device.

**Table 1:** Markers corresponding names.

Marker number	Names
1	R. Clavicle
2	C7
3	R. Shoulder
4	R. Bicep
5	E. Elbow lateral
6	R. Forearm
7	R. Radius
8	R. Hand
9	R. Ulna
10	R. Elbow medial

## Data Availability

The human-device integrated model data used to support the findings of this study have not been made available because the device was only available at our laboratory.
